# Development of Green UV-Vis Method for Direct Determination of Total Sugars in the Aqueous Extract of Teff (*Eragrostis tef* (Zuccagni) Trotter) Grains and Other Cereals

**DOI:** 10.1155/2022/5129510

**Published:** 2022-11-01

**Authors:** Hagos Yisak, Hagos Tukue, Mesfin Redi-Abshiro, Bhagwan Singh Chandravanshi, Estifanos Ele Yaya

**Affiliations:** Department of Chemistry, College of Natural and Computational Sciences, Addis Ababa University, P.O. Box 1176, Addis Ababa, Ethiopia

## Abstract

There is no ultraviolet visible (UV-Vis) spectrophotometric method for the direct determination of total sugars in the aqueous extract of teff grain samples. Therefore, the objective of this study was to develop a green UV-Vis spectrophotometric method to determine total sugars in the aqueous extract of white teff, brown teff, white rice, and red wheat grain samples. The calibration curve was established in the range of 20.11–7,907 mg/L using sucrose as a standard with *R*^2^ = 0.9996. The limit of detection and limit of quantification were 4.4 and 14.6 mg/L, respectively. The relative standard deviation (6.9%) of the method for the sucrose standard was within the acceptable range indicating that the method is precise. The amount of total sugars determined in the white teff (5.48–9.44% (w/w), brown teff (6.17–10.32% (w/w)), white rice (3.19% (w/w)), and red wheat (9.22% (w/w)) grain samples was comparable with other reported cereal grains. Furthermore, the accuracy of the developed analytical method was also evaluated by spiking the known amount of the sucrose standard solution to the white teff, brown teff, white rice, and red wheat sample extracts, and percentage recoveries found were in the acceptable range (85 ± 2 − 105 ± 4%) with an average recovery of 93%, confirming that the new green method is quantitatively reproducible. Hence, a fast, simple, inexpensive, widely used, selective, sensitive, precise, and accurate green UV-Vis method was developed and validated for the direct determination of total sugars in the aqueous extract of teff, white rice, and red wheat grain samples.

## 1. Introduction

Whole grains provide a complete package of health benefits, in contrast to refined grains, which are stripped of essential nutrients in the purification process [1, 2]. Based on World Health Organization's (WHO) reports for 2012 to 2016, consumption of whole grains may decrease the risk of noncommunicable diseases like type 2 diabetes, cardiovascular diseases, cancer, and obesity [2, 3]. Whole grains can help to maintain pancreatic function by increasing glucose-stimulated insulin production in overweight/obese people at risk of type 2 diabetes [4]. Whole grains are invaluable sources of carbohydrates, proteins, fibers, phytochemicals, minerals, and vitamins [2, 5]. The slow release of carbohydrate constituents was found to be useful for diabetic patients [6]. Furthermore, those who consume whole grains live a healthier lifestyle in general, including smoking less, taking less alcohol, and being more physically active [7]. Functional foods obtained from cereals help our body to boost immunity, defend against blood pressure, cholesterol levels, and blood sugar levels, decreasing risk of getting heart failure [5].

Cereals essentially consist of high proportions of carbohydrates, most come from starch and lower proportions come from total sugars [8]. Carbohydrates are important food components affecting taste and nutrition and are the main source of energy in cereals [8, 9]. Teff is a whole grain and superior to other cereals due to being naturally gluten free and is the dominant source of nutrients like carbohydrates, amino acids, minerals, dietary fibers, proteins, dietary polyphenols, starch, and vitamins [6, 10–12]. Volatiles like aldehydes, ketones, and alcohols [12] are rich in unsaturated fatty acids like linoleic, oleic, and linolenic acids [12, 13]. Total carbohydrate is the total of monosaccharides, disaccharides, oligosaccharides, and polysaccharides. Though the total carbohydrate content of teff may vary in different ecology, studies have reported its content to be in the range of 57–86 %w/w [11]. The atherogenicity and thrombogenicity indices used to determine the lipid quality of the white and brown teff grain samples have indicated excellent status of grains compared to other cereal grains, which are useful for human nutrition and health [14]. Teff is a nutritious food even better than the major western staple cereals such as wheat, rice, oats, and barley, which is preferable for celiac disease patients and other types of gluten sensitivity as it is consumed as a whole grain [13, 15, 16].

Sugars are the building blocks of carbohydrates, and they are naturally found in many foods such as cereals, fruits, milk, and vegetables [17]. The term “sugar” in chemistry refers to mono-, di-, and lower oligosaccharides and as the number of monosaccharide units in a molecule increases beyond 2, the sweet taste is considerably less pronounced [18]. This is due to the fact that sugar content of a food item is defined as the sum of monosaccharides and disaccharides [19]. The primary function of sugars in food products is to provide sweetness and energy. Besides, sugars play a very important role in preservation, fermentation, color, and texture in food [17]. Contrary to the advantages of sugars in cereal grains, overconsumption of sugars can result in diarrhea and disturb the blood sugar level. Thus, reporting accurate information to consumers about the quantity of sugars present in various cereal food items is really essential [19].

Sugar analysis forms part of quality control in the food industry to guarantee optimal sugar intake [20]. Because of this reason, several analytical methods were developed and applied for the detection of sugars in different cereal food items. Ion chromatography interfaced with a pulsed amperometric detector (IC-PAD) was used for the simultaneous determination of soluble sugars in both husked and milled rice samples [21]. High-performance anion exchange chromatography with a pulsed amperometric detector (HPAEC-PAD) method has been successfully developed and validated for the simultaneous identification and quantification of sugars in wheat flours [20]. Fourier transform infrared spectroscopy (FT-IR), nuclear magnetic resonance spectroscopy (NMR), and colorimetric methods were also employed to determine sugars [22]. In addition, capillary electrophoresis coupled with electrospray ionization-tandem mass spectrometry (CE-ESI-MS/MS) was applied for the determination of monosaccharides in the corn sample using inositol as an internal standard [23]. High-performance liquid chromatography with an evaporative light scattering detector (HPLC-ELSD), liquid chromatography with mass spectrometry (LC-MS), high-performance liquid chromatography with a refractive index detector (HPLC-RID), and gas chromatography with mass spectrometry (GC-MS) methods were applied to determine sugars in many cereals and seed plants [19].

The majority of the reported analytical methods necessitate the use of carcinogenic organic solvents for extraction, time-consuming sample preparation procedures, multiple chromatographic steps, highly skilled technicians, and high price, making them inconvenient [24]. Among the colorimetric methods for sugar analysis, the phenol-sulfuric acid method is so far the most reliable method and has been extensively used in a wide range of fields. However, it has some serious drawbacks. The coloring agent used in this method, phenol, is not environmentally friendly which poses multiple health hazards. Phenol and its vapors are corrosive to the skin, eye, and respiratory system. Repeated and prolonged contact with the skin can cause dermatitis or second-degree and third-degree burns. Similarly, prolonged or repeated inhalation of phenol vapors causes lung edema. Long-term exposure to phenol also has serious impacts on the central nervous system (it is a strong neurotoxin), kidneys, and liver [22]. Besides, determination of total sugars in cereal grains using sulfuric acids may cause degradations of forming monosaccharides in the presence of hot concentrated acid, which finally results in decreasing the sugar content in the sample [25].

Spectroscopic methods are getting more attention due to their rapidity, cost effectiveness, simplicity, precision, reproducibility, and ability to measure multiple components without tedious sample preparation. In addition, these methods are vastly applicable to determine food composition because of their suitability on direct routine analysis [24]. To the best of the researchers' knowledge, there was no study conducted and reported about the total sugar content in the aqueous extract of cereal grains and other foodstuff using the UV-Vis method. Therefore, to address concrete information to consumers about the quantity of total sugars present in the white, brown teff, white rice, and red wheat grain samples, development of the green chemistry UV-Vis method was found to be very crucial. Hence, the objectives of the study were to (1) optimize the suitable UV-Vis measurement parameters, (2) develop and validate the green UV-Vis method for the direct determination of total sugars in the aqueous extract of white, brown teff, white rice, and red wheat grain samples, and (3) compare the total sugar contents determined in two teff varieties, white rice, and red wheat grain samples with the other commonly used cereal grains.

## 2. Materials and Methods

### 2.1. Apparatus and Instrument

The electronic balance (ARA520, China), grinder (high-speed multifunctional grinder, Shanghai, China), and centrifuge (model: 80–2, China) were used to conduct the experiment. A UV-Vis-NIR spectrometer (Lambda 950, Perkin Elmer, UK) with a 1 cm path length quartz cuvette was used for measuring the absorbance of the prepared standards and sample extracts.

### 2.2. Chemicals

The sucrose standard (Analytical Grade, Guandong Guanghua, Chemical factory, China) was used as received. Distilled water was used as a solvent throughout the study.

### 2.3. Sample Collection and Pretreatment

Fourteen (14) teff samples were collected from the Minjar Shenkora district (North Shewa zone), Were Ilu district (South Wollo zone) of the Amhara region, Ada'a, Bishoftu, and Gimbichu districts (East Shewa zone) of the Oromia region, and Soro and Gomibora districts (Haddiya zone) of the Southern Nations Nationalities and Peoples Region (SNNPR) of Ethiopia The selected areas are the major teff producing areas in the country. The two varieties of teff samples (white and brown teff) were collected from 18, December 2020, to 18, January 2021, from local markets. Besides, to compare the amount of total sugars in teff grains with other cereal grains, wheat (red) and rice (white) samples were collected on June 14/2022 from Sebeta town, which is located 25 km southwest of Addis Ababa. It is a separate district in the Oromia special zone surrounding Addis Ababa city. All samples (Table 1) of each 500 g were collected and stored in a plastic bag under airtight conditions at room temperature. As soon as the samples were transferred to the laboratory, contaminations, like straw, soil, husk, immature seeds, and dust particles, were removed by using a sieve and ground by using an electronic grinder to mesh size 300 *µ*m and then made ready for extraction.

### 2.4. Extraction of Total Sugars in the White and Brown Teff Samples and Other Cereal Grains

To extract the total sugar contents in two teff varieties and other cereal grains (white rice and red wheat), the adapted method reported by Huang et al. [26] was used. In brief, 0.5 g of ground teff, wheat, and rice samples was extracted for 10 min using hot water (65 ± 5°C) by hand shaking, and the mixture was centrifuged for 10 min at 3000 rpm. The supernatant was filtered using Filter Lab filter paper. Then, to determine the total sugar content, a 0.5 mL aliquot of the sample extract was taken and diluted to 40 mL of distilled water. Finally, the diluted sample extract was directly scanned by using a UV-Vis spectrophotometer in the spectral range of 210–182 nm, slit width (1 nm), data interval (0.5 nm), and response time (5 s). The sample preparation up to scanning of the extract was very short, which included only dissolution of powdered cereal grains in water followed by centrifugation and filtration. Results were presented as a mean ± SD from duplicate measurements.

### 2.5. Preparation of Standard Solution

To prepare the sucrose standard for the determination of total sugar contents, 0.2859 g of the sucrose standard was measured using a digital analytical balance and transferred into to a 100 mL volumetric flask. Then, distilled water was added to dissolve the standard, and the measured solution was 36.16 g. The calculated serially diluted solutions were 7,907, 2,860, 894.8, 384.4, 252.8, 49.89, and 20.11 mg/L, respectively. The working standard solutions were scanned in the spectral range (182–210 nm) of the method. The absorption spectral data were collected from their typical absorption peak maximum obtained at 189 nm for plotting calibration curves.

### 2.6. Optimization of Measurement Parameters

In UV-Vis spectrophotometry, changing measurement parameter settings, such as the slit width, scan speed, data interval, and response time, can simultaneously change the width of peaks and noise levels in resulting absorption spectra. Therefore, the optimal parameter settings for the given spectral measurement need to be specified. Hence, the slit width and the response time were optimized in the present study. All the spectral data were collected reasonably in a dark room in order to minimize the noise level.

### 2.7. Validation of the Proposed Method

Validation of the method is an integral part of quality assurance. Good analytical practice cannot be achieved without validation. Method validation is used to ensure that the analytical technique used for a particular test is sufficient for its intended use [27]. In the present study, the analytical method was validated for regression coefficient (*R*^2^), concentration ranges, specificity/selectivity, precision, accuracy, and sensitivity. The regression coefficient (*R*^2^) was evaluated with respect to the measured concentration ranges (20.11–7,907 mg/L). The specificity/selectivity assay was conducted by overlapping absorption spectra of the sucrose standard and sample extract scanned in the method. Precision was determined from repetitive measurements of the lower end of the concentration ranges of the sucrose standard (*n* = 6). Reproducibility (accuracy) was estimated by the standard addition method. The sucrose standard solution was added into the sample extract, and absorption of spiked and unspiked samples was measured. Then, recovery (%R) was calculated using the formula (spiked–unspiked)/amount added) ×100. To measure the sensitivity of the method, the limit of detection (3 × SD) and limit of quantification (10 × SD) [28] were determined by computing the standard deviation (SD) of the blank measurement response (*n* = 6).

## 3. Results and Discussion

### 3.1. Optimization of Measurement Parameters

The slit width is a measurement parameter that specifies the width of the opening through which extent of light enters and exits the monochromator used in a UV-Vis spectrophotometer. As can be seen in Figures 1 and 2, the slit width was optimized at 0.5, 1, 2, 3, and 4 nm at a fixed data interval (0.5 nm) and response time (0.52 s) using the sucrose standard (4.9% w/w). As can be observed in Figure 1, the peak absorbance decreases with an increasing slit width, which is attributed to the emergence of light intensity that may have not passed through the sample. Excessively decreasing the slit width affects the sensitivity due to the exponentially increasing reflection loss of light intensity at a shorter wavelength that arises from increased dispersion phenomena. Therefore, the response time was increased almost ten-fold of 0.52 s to 5 s to suppress the noise level and consequently improve the sensitivity of the proposed method. Hence, the optimum slit width used throughout the experimental work was 1 nm since the peak absorbance was almost the same with the slit width at 0.5 nm (Figure 2). Besides, an optimized response time of 5 s was used to collect the desired experimental data.

### 3.2. Evaluation of Analytical Parameters of the Proposed Green UV-Vis Method

Analytical parameters of the newly developed green UV-Vis method for the determination of total sugars were evaluated in terms of regression coefficient, limit of detection (LOD), limit of quantification (LOQ), specificity, precision, and accuracy (recovery). The overlay spectra of the sucrose standard is shown in Figure 3, while the calibration curve equation (Figure 4) established for the sucrose standard was *y* = −1.2949 × 10^−8^*x*^2^ + 0.00031*x* + 0.02988, where *y* and *x*, respectively, represent peak absorbance and concentration of sucrose in mg/L. The magnitude of the regression coefficient (*R*^2^ = 0.9996) indicated that there is a strong correlation between the concentration and response in the measured concentration range of 20.11–7.907 mg/L for sucrose. The LOD and LOQ of the developed method were 4.4 mg/L and 14.6 mg/L, respectively, indicating that the method is sensitive which could be able to detect small amount of the desired analyte. The ability of the analytical method to reliably measure the total amount of sugars in the presence of interferences that may be present in the samples matrix was evaluated by overlapping the spectra of sucrose, glucose, fructose, and maltose standards and sample extracts. To further validate the specificity/selectivity of the proposed method, four sugar standards (glucose, fructose, sucrose, and maltose) standards were scanned and overlapped so that the region could be selective for the direct determination of total sugars in intended cereal grains (Figure 5). Besides, the precision of the method was evaluated by scanning the lower end of the calibration curve's concentration six times and calculating the relative standard deviation (RSD), and the result found was 6.9%, which confirms that the proposed method is repeatable. Furthermore, the accuracy of the developed analytical method was also evaluated by spiking the known amount of the sucrose standard solution to the real sample extracts (white teff, brown teff, white rice, and red wheat), and percentage recoveries found were in the acceptable range of 85 ± 3–105 ± 4%. The recovery result (Table 2) has assured that the method is reliably reproducible.

### 3.3. Application of the Newly Developed Green UV-Vis Method for Determination of Total Sugars in the Aqueous Extract of Teff and Other Cereal Grains

The amount of total sugars in the aqueous extract of white and brown teff, white rice, and red wheat grain samples were determined by scanning the sample extract in the range of 182–210 nm, with a slit width of 1 nm, data interval of 0.5 nm, and response time of 5 seconds. The total sugar content in the intended cereal samples was calculated using the calibration equations by further considering the dilution factor and was reported as grams of sucrose equivalent per 100 g (%w/w) of white teff, brown teff, white rice, and red wheat flour on dry basis. The content of total sugars (Table 3) in the white and brown teff samples ranged between 5.48 and 9.44% (w/w) and 6.17–10.32% (w/w), respectively. Furthermore, the other common cereal grains (white rice and red wheat) (Figure 6) were also determined for comparison purposes. The contents of white rice (3.19 ± 0.24%) and red wheat (9.22 ± 0.20%) were determined. The content of total sugars found in teff (white and brown) was comparable with the amount of total sugars determined in red wheat grain but higher than the white rice grain sample.

Results of the present study are in agreement with the content of total sugars in wheat (7.8 %w/w) [29]. However, it is higher than the maize (3.66 %w/w), sorghum (2.56 %w/w), and millet (3.31 %w/w), determined by using the phenol-sulfuric acid-based UV-Vis method [8], and rye (2.3 %w/w) [29]. Furthermore, the total sugar content in rice samples determined by the sulfuric acid, UV-Vis method was reported by Omar et al. [25], whichis in the range of 7.93–23.34%, which is higher than that of the present study. Omar et al. [25] stated that the sulfuric acid method may cause degradations of forming monosaccharides in the presence of hot concentrated acid, which finally results in decreasing the sugar content in the sample. It might be because of this reason that the amount of total sugars in most cereal grains determined by the sulfuric acid method is lowered.

## 4. Conclusion

A simple, fast, cost-effective, selective, widely used, sensitive, repeatable, and reproducible green UV-Vis method was developed and validated for the first time to directly determine the total amount of sugars in the aqueous extract of white teff, brown teff, white rice, and red wheat grain samples. The total sugar contents in the intended cereal grains were successfully determined by the developed method, and the results were comparable with the reported literature. The differences in content of total sugars in the cereal grains might be due to the variations in their cultivars, varieties, types of soil, and their geographical locations. The proposed method has, therefore, the advantage over other methods as it avoids use of phenol, sulfuric acid, and other organic solvents. The sample preparation up to scanning of the extract was very short, which included only dissolution of powdered white teff, brown teff, white rice, and red wheat grains in water followed by centrifugation and filtration. Hence, the new green UV-Vis method can be suitable and applicable for the routine analysis of total sugars in any foodstuff and is safe for health and eliminates environmental hazards.

## 5. Recommendations

Findings of this study could be very useful for consumers to be aware of the nutritional value of water-soluble total sugars of white teff, brown teff, white rice, and red wheat grains. However, the comprehensive study should be conducted by collecting more samples from different regional parts of Ethiopia, and statistical tools like PCA, LDA, and PLS should be employed to differentiate cereal grains based on the water-soluble total sugar contents using the newly developed green UV-Vis method. Furthermore, the soil type, rainfall, temperature, and quality of irrigation water should be considered during analysis.

## Figures and Tables

**Figure 1:** Overlay of absorption spectra of the sucrose standard (4.9 %w/w) dissolved in water and scanned at different slit widths and response time (0.52 seconds).

**Figure 2:** Graph of peak absorbance versus slit width of the sucrose standard (4.9 %w/w) dissolved in water.

**Figure 3:** Overlay of absorption spectra of different concentrations of the sucrose standard dissolved in water.

**Figure 4:** Calibration curve of the sucrose standard dissolved in water.

**Figure 5:** Normalized absorption spectra of the four sugar standards dissolved in water.

**Figure 6:** Normalized absorption spectra of the sucrose standard dissolved in water and total sugars in the white teff, brown teff, white rice, and red wheat samples extracted in water.

**Table 1:** Sampling areas and sample ID of the white and brown teff grains (*Eragrostis tef* (Zuccagni) Trotter), white rice, and red wheat varieties cultivated in Ethiopia.

Regions	Administrative zones	Districts	Variety of cereals	Sample ID
Amhara	North Shewa	Minjarna Shenkora	White teff	AW-1
			Brown teff	AB-19
	South Wollo	Were Ilu	White teff	AW-6
			Brown teff	AB-24

Oromia	East Shewa	Ada'a	White teff	OW-13
			Brown teff	OB-31
		Bishoftu	White teff	OW-14
			Brown teff	OB-32
		Gimbichu	White	OW-15
			Brown	OB-33
	South West Shewa	Sebeta	White rice	WR-01
			Red wheat	RWh-02

SNNPR	Hadiya	Soro	White teff	SW-17
			Brown teff	SB-35
		Gomibora	White teff	SW-18
			Brown teff	SB-36

ID, identification.

**Table 2:** Recovery results of total sugars determined by the newly developed green UV-VIS method.

Variety of samples	Trial	Amount of total sugar in the sample before spiking (mg/L)	Amount of sucrose spiked (mg/L)	Amount of total sugars found after spiking (mg/L)	Recovery (%)	Mean recovery (%)
White teff	1	672.50	107.6	762.89	83.7	86 ± 2
	2	690.63	107.6	784.24	86.7	

Brown teff	1	604.52	107.6	713.56	100.96	105 ± 4
	2	617.61	107.6	733.50	107.31	

Red wheat	1	240.5	96.2	276.6	93.8	95 ± 2
	2	245.5	96.2	282.7	96.6	

White rice	1	269.6	96.2	301.6	83.1	85 ± 3
	2	270.5	96.2	303.9	86.8	

**Table 3:** Amount of total sugars (mean ± SD) in white and brown teff (*Eragrostis tef* (Zuccagni) Trotter), white rice, and red wheat grains determined by the newly developed UV-VIS method.

Regions	Variety of cereals	Sample ID	Total sugars (%w/w)
Amhara	White teff	AW-1	8.30 ± 0.48
	Brown teff	AB-19	7.46 ± 0.25
	White teff	AW-6	7.63 ± 0.53
	Brown teff	AB-24	8.97 ± 0.19

Oromia	White teff	OW-13	7.97 ± 0.26
	Brown teff	OB-31	10.32 ± 0.34
	White teff	OW-14	9.08 ± 0.30
	Brown teff	OB-32	8.47 ± 0.50
	White	OW-15	9.44 ± 0.53
	Brown	OB-33	8.21 ± 0.38
	White rice	WR-01	3.19 ± 0.24
	Red wheat	RWh-02	9.22 ± 0.20

SNNPR	White teff	SW-17	5.94 ± 0.33
	Brown teff	SB-35	6.17 ± 0.11
	White teff	SW-18	5.48 ± 0.21
	Brown teff	SB-36	7.47 ± 0.24

ID, identification.

## Data Availability

All the data are included in the manuscript.
